The article "Stochastic Stability Analysis for Stochastic Coupled Oscillator Networks with Bidirectional Cross-Dispersal" was published in 2022. Journal: Comput Intell Neurosci.

# Stochastic Stability Analysis for Stochastic Coupled Oscillator Networks with Bidirectional Cross-Dispersal

**DOI:** 10.1155/2022/2742414

**Published:** 2022-06-08

**Authors:** Xiaoqi Liu, Shang Gao

**Affiliations:** Department of Mathematics, Northeast Forestry University, Harbin 150040, China

## Abstract

It is well known that stochastic coupled oscillator network (SCON) has been widely applied; however, there are few studies on SCON with bidirectional cross-dispersal (SCONBC). This paper intends to study stochastic stability for SCONBC. A new and suitable Lyapunov function for SCONBC is constructed on the basis of Kirchhoff's matrix tree theorem in graph theory. Combining stochastic analysis skills and Lyapunov method, a sufficient criterion guaranteeing stochastic stability for the trivial solution of SCONBC is provided, which is associated with topological structure and coupling strength of SCONBC. Furthermore, some numerical simulation examples are given in order to illustrate the validity and practicability of our results.

## 1. Introduction

In the past few decades, stochastic coupled oscillator network (SCON) has attracted extensive attention from the scientific community and has been widely used in many fields, such as physics [1–3], biology [4, 5], engineering [6, 7], and so on. On the other hand, dispersal is a common phenomenon in nature, which is due to the imbalance of oscillators in different regions. A lot of results about single dispersal have appeared in [8–10] since it plays an important role in the research of application problems. In addition, it is worth noting that dispersal also occurs between different oscillators of different groups, that is, bidirectional cross-dispersal. To the best of the authors' knowledge, SCON with bidirectional cross-dispersal (SCONBC) is rarely studied. Based on the above discussion, the purpose of this paper is to research the stochastic stability of SCONBC.

As is known to all, the Lyapunov method is a powerful tool for analyzing the stochastic stability of SCONBC. For all that, owing to the complex structure of stochastic coupled oscillator networks with bidirectional cross-dispersal terms, it is quite challenging to construct the Lyapunov function for SCONBC. Li et al. proposed a method to solve this problem by combining graph theory in [11]. In this paper, inspired by them, we successfully construct a suitable Lyapunov function for SCONBC by the approach combining Kirchhoff's matrix tree theorem in graph theory, which solves the above problem we mentioned and has been applied in various articles [12, 13].

Gao et al. has researched periodic solutions for neutral coupled oscillator network with feedback and time-varying delay and the existence of periodic solutions for discrete-time coupled systems on networks with time-varying delay in [14, 15]. Compared with the existing literature, our innovations and contributions are as follows:

1. Bidirectional cross-dispersal terms are taken into SCONBC, and a new Lyapunov function for SCONBC is constructed by applying Kirchhoff's matrix tree theorem in graph theory.
2. A sufficient criterion is obtained, which combines stochastic analysis skills and can show how topological structure and coupling strength affect the stochastic stability for the trivial solution of SCONBC.
3. Some numerical examples and their simulation results are provided to validate the applicability of our theoretical results.

The structure of this paper is arranged as follows. Some necessary notations are given in Section 2.1, and concepts about graph theory are provided in Section 2.2. In Section 3, we establish SCONBC and give its model formulation. A sufficient criterion ensuring stochastic stability for the trivial solution of SCONBC and its proof is offered in Section 4.  Section 5 provides some numerical simulation examples. Finally, the conclusion is drawn in Section 6.

## 2. Preliminary

### 2.1. Notations

Throughout this paper, the notations in Table 1 will be used unless otherwise specified.

Other notations will be explained where they first appear.

### 2.2. Graph Theory

Here, we introduce some useful concepts associated with graph theory. A digraph *𝒢*=(*𝔸*, *E*) contains a set *𝔸*={1,2,…, *n*} of vertices and a set *E* of arcs (*k*,  *h*) which lead from initial vertex *k* to terminal vertex *h*, and each vertex of digraph *𝒢* is regarded as an oscillator. Define the weight matrix of *𝒢* as *Q*=(*q*_*kh*_)_*n*×*n*_, where *q*_*kh*_ > 0 if there exists an arc from vertex *h* to vertex *k*. Digraph *𝒢* with the weighted matrix *Q* is denoted by (*𝒢*, *Q*). The Laplacian matrix of digraph (*𝒢*, *Q*) is defined as

(1) $$\begin{array}{c} L=\left(\begin{array}{cccc} \sum_{i\neq 1}q_{1i} & -q_{12} & \cdots & -q_{1n}\\ -q_{21} & \sum_{i\neq 2}q_{2i} & \cdots & -q_{2n}\\ \vdots & \vdots & \ddots & \vdots \\ -q_{n1} & -q_{n2} & \cdots & \sum_{i\neq n}q_{ni} \end{array}\right). \end{array}$$

For other details on graph theory, we refer the readers to [16, 17].

At the end of this section, we provide a lemma in graph theory.

**Lemma 1 .**

(see [16]) (Kirchhoff's matrix tree theorem). Assume that *n* ≥ 2. Let *q*_*k*_ denote the cofactor of the *k*-th diagonal element of the Laplacian matrix of the weighted digraph (*𝒢*, *Q*). Then,

(2) $$\begin{array}{c} q_{k}=\sum_{T\in T_{k}}W\left(T\right),\;k\in K, \end{array}$$

where *𝕋*_*k*_ is the set of all spanning trees *𝒯* of the weighted digraph (*𝒢*, *Q*) that are rooted at vertex *k* and *W*(*𝒯*) is the weight of *𝒯*. Particularly, if the weighted digraph (*𝒢*, *Q*) is strongly connected, then *q*_*k*_ > 0.

## 3. Model Formulation

Stochastic oscillators have important applications in many branches of industry [18], such as biology [19], physics [20], and so on. In this section, we provide a detailed description of SCONBC. Let us firstly see the stochastic oscillator equation with white noise, which is expressed as

(3) $$\begin{array}{c} \ddot{x}\left(t\right)+\alpha \dot{x}\left(t\right)=\beta x\left(t\right)\dot{Β}\left(t\right), \end{array}$$

where *x*(*t*) ∈ ℝ^*n*^ is the system state, *α* and *β* are damping coefficients, and *Β*(*t*) is a one-dimensional Brownian motion. In this paper, we consider *n*  oscillators and the *k*-th oscillator is denoted as follows:

(4) $$\begin{array}{c} {\ddot{x}}_{k}\left(t\right)+\alpha_{k}{\dot{x}}_{k}\left(t\right)=\beta_{k}x_{k}\left(t\right)\dot{Β}\left(t\right),\;k\in K, \end{array}$$

where *x*_*k*_(*t*) ∈ ℝ denotes the system state of the *k*-th oscillator. Since the bidirectional cross-dispersal is a common phenomenon in our real life, in order to describe the dynamic behavior of system (3) more accurately, the bidirectional cross-dispersal terms are added, and based on a transform of $y_{k}\left(t\right)={\dot{x}}_{k}\left(t\right)$, system (4) can be written as follows:

(5) $$\begin{array}{c} \left\{\begin{array}{c} \text{d}x_{k}\left(t\right)=\left[y_{k}\left(t\right)+\sum_{h=1}^{n}a_{kh}\left(y_{h}\left(t\right)-x_{k}\left(t\right)\right)\right]\text{ d}t,\\ \text{d}y_{k}\left(t\right)=\left[-\alpha_{k}y_{k}\left(t\right)+\sum_{h=1}^{n}b_{kh}\left(x_{h}\left(t\right)-y_{k}\left(t\right)\right)\right]\text{d}t+\beta_{k}x_{k}\left(t\right)\text{d}Β\left(t\right),\;k,h\in K, \end{array}\right. \end{array}$$

where the dispersal of *y*(*t*) in the *h*-th group of oscillators which is from *x*(*t*) in the  *k*-th group of oscillators is expressed as the function *a*_*kh*_(*y*_*h*_(*t*) − *x*_*k*_(*t*)) and the function *b*_*kh*_(*x*_*h*_(*t*) − *y*_*k*_(*t*)) denotes the dispersal of *x*(*t*) in the *h*-th group of oscillators which is from *y*(*t*) in the *k*-th group of oscillators. *a*_*kh*_ and *b*_*kh*_ represent the coupling strength of the irreducible coupling configuration matrices *A*=(*a*_*kh*_)_*n*×*n*_ and *B*=(*b*_*kh*_)_*n*×*n*_, separately. Specially, it is worth noting that *a*_*kh*_ and *b*_*kh*_  = 0 if there is no cross-dispersal from *x*(*t*) in the *k*-th group of oscillators to *y*(*t*) in the *h*-th group of oscillators and from *y*(*t*) in the *k*-th group of oscillators to *x*(*t*) in the *h*-th group of oscillators.

The form of SCONBC (5) is too complex for the readers to read and will make subsequent proof tedious; therefore, we solve these problems by simplifying SCONBC (5) into the following SCONBC (6):

(6) $$\begin{array}{c} dz_{k}\left(t\right)=f_{k}\left(z_{k}\left(t\right),t\right)dt+g_{k}\left(z_{k}\left(t\right),t\right)dΒ\left(t\right), \end{array}$$

where

(7) $$\begin{array}{c} z_{k}={\left(x_{k},y_{k}\right)}^{Τ},g_{k}={\left(0,\beta_{k}x_{k}\right)}^{Τ}, \end{array}$$

(8) $$\begin{array}{c} f_{k}\left(z_{k},t\right)={\left(y_{k}+\sum_{h=1}^{n}a_{kh}\left(y_{h}-x_{k}\right),-\alpha_{k}y_{k}+\sum_{h=1}^{n}b_{kh}\left(x_{h}-y_{k}\right)\right)}^{Τ}. \end{array}$$

We let the initial value *z*(0)=*z*_0_, and it is easy to see that there exists a trivial solution denoted as *z*(*t*; *z*_0_, 0)=*z*(*t*) to SCONBC (4).

Subsequently, for any *V*(*z*, *t*) ∈ *C*^2,1^(ℝ^*n*^ × ℝ^+^; ℝ^+^), a differential operator of SCONBC (4) ℒ*V* is normally defined by [18]

(9) $$\begin{array}{c} ℒV\left(z,t\right)≜\frac{\partial V\left(z,t\right)}{\partial t}+\frac{\partial V\left(z,t\right)}{\partial z}f\left(z,t\right)+\frac{1}{2}\text{trace}\left[{\left(g\left(z,t\right)\right)}^{Τ}\frac{\partial^{2}V\left(z,t\right)}{\partial z^{2}}g\left(z,t\right)\;\right]. \end{array}$$

Our purpose is to explore the stochastic stability for the trivial solution of SCONBC (4) in this paper, and its definition is given as follows.

**Definition 1 .**

If for every *ε* ∈ (0,1), *t* ∈ ℝ^+^ and the constant *τ* > 0, there exists *δ*=*δ*(*z*_0_, *ε*, *τ*) > 0 such that

(10) $$\begin{array}{c} \mathbb{P}\left\{\left|z\left(t\right)\right|<\tau ,t\geq 0\right\}\geq 1-\varepsilon , \end{array}$$

for the initial value |*z*_0_| < *δ*, then the trivial solution of SCONBC (3) is stochastically stable.

## 4. Main Results

In this section, we will provide a theorem and its proof in regard to the stochastic stability for the trivial solution of SCONBC (4).

**Theorem 1 .**

The trivial solution of SCONBC (4) is stochastically stable if the following condition is satisfied for any *k*, *h* ∈  *𝕂*.

(11) $$\begin{array}{c} c_{k}+d_{k}\beta_{k}^{2}\leq \sum_{h=1}^{n}\left(c_{k}a_{kh}-{\text{d}}_{k}b_{kh}\right)\leq 2\alpha_{k\;}{\text{d}}_{k}-c_{k}, \end{array}$$

where *c*_*k*_  and *d*_*k*_ are the cofactors of the *k*-th diagonal element of the Laplacian matrix in digraphs (*𝒢*, *A*) and (*𝒢*, *B*), respectively.

**Proof**

We firstly construct a Lyapunov function as follows:

(12) $$\begin{array}{c} V\left(z,t\right)=\sum_{h=1}^{n}c_{k}x_{k}^{2}+\sum_{k=1}^{n}{\text{d}}_{k}y_{k}^{2}, \end{array}$$

where *c*_*k*_, *d*_*k*_ > 0 in light of Lemma 1.

According to the differential operator defined above, it can be obtained that

(13) $$\begin{array}{c} ℒV\left(z,t\right)=\left(2\sum_{k=1}^{n}c_{k}x_{k},2\sum_{k=1}^{n}d_{k}y_{k}\;\right)\left(\begin{array}{c} y_{k}+\sum_{h=1}^{n}a_{kh}\left(y_{h}-x_{k}\right)\\ -\alpha_{k}y_{k}+\sum_{h=1}^{n}b_{kh}\left(x_{h}-y_{k}\right) \end{array}\right),+\frac{1}{2}\left(0,\beta_{k}x_{k}\right)\left(\begin{array}{cc} 2\sum_{k=1}^{n}c_{k} & 0\\ 0 & 2\sum_{k=1}^{n}{\text{d}}_{k} \end{array}\right)\left(\begin{array}{c} 0\\ \beta_{k}x_{k} \end{array}\right),\\ \leq \sum_{k=1}^{n}c_{k}\left\{\left(x_{k}^{2}+y_{k}^{2}\right)+\sum_{k=1}^{n}a_{kh}\left[H_{kh}^{\left(1\right)}\left(y_{k},y_{h},t\right)+y_{k}^{2}-x_{k}^{2}\right]\right\}+\sum_{k=1}^{n}d_{k}\left\{-2\alpha_{k}y_{k}^{2}+\sum_{k=1}^{n}b_{kh}\left[H_{kh}^{\left(2\right)}\left(x_{k},x_{h},t\right)+x_{k}^{2}-y_{k}^{2}\right]\right\}+\sum_{k=1}^{n}d_{k}\beta_{k}^{2}x_{k}^{2}, \end{array}$$

where *H*_*kh*_^(1)^(*y*_*k*_, *y*_*h*_, *t*)=*y*_*h*_^2^ − *y*_*k*_^2^ and *H*_*kh*_^(2)^(*x*_*k*_, *x*_*h*_, *t*)=*x*_*h*_^2^ − *x*_*k*_^2^. In accordance with combination identical equation in graph theory (see [11], Theorem 2.2) and the fact *W*(𝒬) ≥ 0 as well as $W\left(\tilde{𝒬}\right)\geq 0$, we can know that

(14) $$\begin{array}{c} \sum_{k,h=1}^{n}c_{k}a_{kh}H_{kh}^{\left(1\right)}\left(y_{k},y_{h},t\right)=\sum_{Q\in \mathbb{Q}}W\left(Q\right)\sum_{\left(k,h\right)\in E\left(C_{Q}\right)}H_{kh}^{\left(1\right)}\left(y_{k},y_{h},t\right)\leq 0, \end{array}$$

(15) $$\begin{array}{c} \sum_{k,h=1}^{n}d_{k}b_{kh}H_{kh}^{\left(2\right)}\left(x_{k},x_{h},t\right)=\sum_{\tilde{Q}\in \tilde{\mathbb{Q}}}W\left(\tilde{Q}\right)\sum_{\left(k,h\right)\in E\left(C_{\tilde{Q}}\right)}H_{kh}^{\left(1\right)}\left(y_{k},y_{h},t\right)\leq 0, \end{array}$$

where ℚ and $\tilde{\mathbb{Q}}$ are the sets of all spanning unicyclic graphs of the weighted digraphs (*𝒢*, *A*) and (*𝒢*, *B*), respectively, *W*(𝒬) and $W\left(\tilde{𝒬}\right)$ are the weights of ℚ and $\tilde{\mathbb{Q}}$ separately, and *𝒞*_*Q*_ and ${𝒞}_{\tilde{𝒬}}$, respectively, denote the directed cycle of ℚ as well as $\tilde{\mathbb{Q}}$. Then, taking inequalities (14) and (15) into inequality (1, we can get

(16) $$\begin{array}{c} ℒV\left(z,t\right)\leq \sum_{k=1}^{n}\left\{\begin{array}{c} \left[c_{k}-\sum_{h=1}^{n}\left(c_{k}a_{kh}-d_{k}b_{kh}\right)+{\text{d}}_{k}\beta_{k}^{2}\right]x_{k}^{2}+\\ \left[c_{k}+\sum_{h=1}^{n}\left(c_{k}a_{kh}-d_{k}b_{kh}\right)-2\alpha_{k}{\text{d}}_{k}\right]y_{k}^{2} \end{array}\right\}\leq 0. \end{array}$$

On the other hand, let *m*=min_1≤*k*≤*n*_{*c*_*k*_, *d*_*k*_}, where *m* is a positive constant and we can get

(17) $$\begin{array}{c} V\left(z,t\right)\geq \sum_{k=1}^{n}m{\left|z_{k}\right|}^{2}\geq m{\left|z\right|}^{2}≜\mu \left(\left|z\right|\right), \end{array}$$

where *μ*(.) ∈ *𝒦*_*∞*_ and *μ*(.)=*m*(.)^2^.  It is obvious that *V*(*z*, *t*) is a continuous positive definite function and *V*(0,0)=0. Hence, for every *ε* ∈ (0,1) and the constant *τ* > 0, we can find a *δ*=*δ*(*z*_0_, *ε*, *τ*) such that

(18) $$\begin{array}{c} \frac{1}{\varepsilon }\underset{z\in S_{\delta }}{\sup}V\left(z,0\right)\leq \mu \left(\tau \right) \end{array}$$

where *S*_*δ*_={*z* : |*z*| < *δ*}. Then, it can be easily obtained that *δ* < *τ*. Subsequently, we let *z*_0_ ∈ *S*_*δ*_ and establish a stopping time sequence *r*=inf{*t* ≥ 0, *z*(*t*) ∉ *S*_*τ*_}, where *S*_*τ*_={*z* : |*z*| < *τ*}.

Based on $\text{It}\hat{\text{o}}$'s formula, we can obtain

(19) $$\begin{array}{c} V\left(z\left(t\Lambda r\right),t\Lambda r\right)=V\left(z_{0},0\right)+\int_{0}^{t\Lambda r}ℒV\left(z\left(s\right),s\right)\text{d}s+\int_{0}^{t\Lambda r}\frac{\partial V\left(z\left(s\right),s\right)}{\partial z}g\left(z\left(s\right),s\right)\text{d}Β\left(s\right). \end{array}$$

Taking the expectation of both sides of equality (19) and on the basis of inequality (16), it is derived that

(20) $$\begin{array}{c} EV\left(z\left(t\Lambda r\right),t\Lambda r\right)\leq V\left(z_{0},0\right)\;. \end{array}$$

When *r* ≤ *t*, in conformity with inequality (17), we can get

(21) $$\begin{array}{c} EV\left(z\left(t\Lambda r\right),t\Lambda r\right)\geq E\left[I_{\left\{r\leq t\right\}}V\left(z\left(r\right),r\right)\right]\geq \mu \left(\tau \right)\mathbb{P}\left\{r\leq t\right\}. \end{array}$$

According to inequalities (20) and (21) and *δ* that we find above, it can be obtained that

(22) $$\begin{array}{c} \mathbb{P}\left\{r\leq t\right\}\leq \varepsilon . \end{array}$$

Let *t*⟶*∞*, and we can get

(23) $$\begin{array}{c} \mathbb{P}\left\{r\leq \infty \right\}\leq \varepsilon . \end{array}$$

Therefore,

(24) $$\begin{array}{c} \mathbb{P}\left\{\left|z\left(t\right)\right|<\tau ,t\geq 0\right\}\geq 1-\varepsilon , \end{array}$$

which means that the trivial solution of SCONBC (4) is stochastically stable according to Definition 1.

**Remark 1 .**

The condition in Theorem 1 is mild and reflects the close relationship between the stochastic stability for the trivial solution of SCONBC (4) and the topological structure of digraphs (*𝒢*,  *A*) and (*𝒢*,  *B*). In addition, due to the high dimension as well as the complex structure of SCONBC (4), it is obviously difficult to establish a suitable Lyapunov function for SCONBC (4). In this paper, we propose a framework method to solve this problem, that is, constructing Lyapunov function by Kirchhoff's matrix tree theorem in graph theory, and the method can be applied to more complex network models.

**Remark 2 .**

In recent years, the dynamic behavior of stochastic coupled oscillator networks has been widely studied and applied. Zhang et.al researched the exponential synchronization problem of stochastic coupled oscillator networks with time-varying delays in [21]. In [22], Li et al. illustrated the synchronous stationary distribution of hybrid stochastic coupled oscillator networks. Different from the above results, this paper explores stochastic coupled oscillators with bidirectional cross-dispersal terms, which makes the study of SCONBC (4) more practical.

## 5. Numerical Test

In this part, some numerical simulation examples are provided to verify the validity of our results. Here, we consider SCONBC (4) with *n*=3 oscillators and let positive constants

(25) $$\begin{array}{c} \alpha_{1}\;=7.33,\alpha_{2}=3.70,\alpha_{3}=6.37,\\ \beta_{1}=1.20,\beta_{2}=0.88,\beta_{3}=0.57. \end{array}$$

The coupling configuration matrices are

(26) $$\begin{array}{c} A=\left(\begin{array}{ccc} 0 & 1.80 & 0.48\\ 1.51 & 0 & 0.32\\ 0.52 & 1.63 & 0 \end{array}\right), \end{array}$$

(27) $$\begin{array}{c} B=\left(\begin{array}{ccc} 0 & 1.05 & 0.12\\ 0.45 & 0 & 0.23\\ 0.24 & 1.21 & 0 \end{array}\right), \end{array}$$

which are irreducible evidently. By calculation, we can get that

(28) $$\begin{array}{c} c_{1}=3.4129,c_{2}=4.6524,c_{3}=1.4544,d_{1}=0.7077,d_{2}=1.6677,d_{3}=0.3231, \end{array}$$

which means that the condition in Theorem 1 is met. Therefore, SCONBC (4) is stochastically stable, whose dynamic behavior can be seen in Figures 1–3 with the initial values as follows:

(29) $$\begin{array}{c} z_{1}={\left(2.00,1.00\right)}^{Τ},z_{2}={\left(-0.20,0.80\right)}^{Τ},z_{3}={\left(1.00,-0.04\right)}^{Τ}. \end{array}$$

## 6. Conclusion

In this paper, we have researched stochastic stability for the trivial solution of SCONBC (4). Based on Kirchhoff's matrix tree theorem in graph theory, a new and suitable Lyapunov function is constructed. A sufficient criterion which ensures that the trivial solution of SCONBC (4) is stochastically stable has been given by applying stochastic analysis skills and Lyapunov method. Finally, some numerical simulation examples have been presented to explain the validity of our theories. Compared with the stochastic coupled oscillator networks studied in the previous papers [14, 15], this paper considers the bidirectional cross-dispersal terms. Due to the phenomenon of bidirectional cross-dispersal between different oscillators in different groups, our results can be widely used in the study of biological populations, the interaction of physical oscillators, and so on. However, this paper has considered the small noise in real life, namely, white noise, but in real life, there are many colored noises such as Levy noise, Poisson noise, second moment process noise, and so on, which is the limitation of this article and our future research work.

## Figures and Tables

**Figure 1:** The sample path of the trivial solution *z*_1_(*t*) for SCONBC (4).

**Figure 2:** The sample path of the trivial solution *z*_2_(*t*) for SCONBC (4).

**Figure 3:** The sample path of the trivial solution *z*_3_(*t*) for SCONBC (4).

**Table 1:** Notations used in this paper.

Notation	Description
ℝ	The set of real numbers
*ℝ* ^*n*^	The set of *n*-dimensional Euclidean space
*ℝ* ^+^	[0, +*∞*)
*Τ*	The transpose of vector
(*Ω*, ℱ, {ℱ_*t*_}_*t*≥0_, ℙ)	A complete probability space
{ℱ_*t*_}_*t*≥0_	A filtration satisfying the usual conditions
ℙ	A probability measure
*𝔼*	The expectation of ℙ
*Β*(*t*)	A one-dimensional Brownian motion defined on the complete probability space
|*z*|	The Euclidean norm of vector $z={\left(z_{1},\cdots z_{n}\right)}^{Τ}\varepsilon {\mathbb{R}}^{n},\;\left|z\right|={\left(\overset{n}{\underset{k}{\sum }}z_{k}^{2}\right)}^{1/2}$
*𝕂*	A collection of {1,2,…, *n*}
*𝒦*_*∞*_	A collection of *μ*(*·*) which is on ℝ^+^⟶ℝ^+^, strictly increasing and unbounded, and *μ*(0)=0
*V*(*z*, *t*)	The family of all nonnegative functions which is on ℝ^*n*^ × ℝ^+^ and is continuously twice differentiable in *z* and once in *t* is represented by *C*^2,1^(ℝ^*n*^ × ℝ^+^; ℝ^+^)
*I*_Λ_	An indicator function, where Λ is a collection; if *tϵ*Λ, *I*_Λ_=1; otherwise, *I*_Λ_=0

## Data Availability

The data used to support the findings of this study are available from the corresponding author upon request.

## References

[1] Li P., Yi Z. (2008). Synchronization of Kuramoto oscillators in random complex networks. *Physica A: Statistical Mechanics and Its Applications*.

[2] Liu Y., Yu P., Chu D., Su H. (2019). Stationary distribution of stochastic Markov jump coupled systems based on graph theory. *Chaos, Solitons & Fractals*.

[3] Pototsky A., Janson N. B. (2009). Delay-induced spatial correlations in one-dimensional stochastic networks with nearest-neighbor coupling. *Physical Review A*.

[4] Bagheri N., Taylor S. R., Meeker K., Petzold L. R., Doyle F. J. (2008). Synchrony and entrainment properties of robust circadian oscillators. *Journal of The Royal Society Interface*.

[5] Lorenzo M. N., Montejo N., Pérez-Muñuzuri V., Pérez-Villar V. (2004). Spatiotemporal behavior in networks of Ca3 region in the hippocampus. *Neurocomputing*.

[6] Liu J., Feng K., Qu Y., Nawaz A. H., Wang F. (2021). Stability analysis of T-S fuzzy coupled oscillator systems influenced by stochastic disturbance. *Neural Computing & Applications*.

[7] Chen B.-S., Hsu C.-Y. (2012). Robust synchronization control scheme of a population of nonlinear stochastic synthetic genetic oscillators under intrinsic and extrinsic molecular noise via quorum sensing. *BMC Systems Biology*.

[8] Liu L., Cai W., Wu Y. (2012). Global dynamics for an SIR patchy model with suspectibles dispersal. *Advances in Differential Equations*.

[9] Wang W., Zhao X.-Q. (2004). An epidemic model in a patchy environment. *Mathematical Biosciences*.

[10] Chen T., Sun Z., Wu B. (2017). Stability of multi-group models with cross-dispersal based on graph theory. *Applied Mathematical Modelling*.

[11] Li M. Y., Shuai Z. (2010). Global-stability problem for coupled systems of differential equations on networks. *Journal of Differential Equations*.

[12] Gao S., Peng C., Li J., Kang R., Liu X., Zhang C. (2022). Global asymptotic stability in mean for stochastic complex networked control systems. *Communications in Nonlinear Science and Numerical Simulation*.

[13] Zhang C., Li W., Wang K. (2014). A graph-theoretic approach to stability of neutral stochastic coupled oscillators network with time-varying delayed coupling. *Mathematical Methods in the Applied Sciences*.

[14] Gao S., Zhou H., Wu B. (2017). Periodic solutions for neutral coupled oscillators network with feedback and time-varying delay. *Applicable Analysis*.

[15] Gao S., Guo H., Chen T. (2019). The existence of periodic solutions for discrete-time coupled systems on networks with time-varying delay. *Physica A: Statistical Mechanics and Its Applications*.

[16] West D. B. (2001). *Introduction to Graph Theory*.

[17] Biggs N., Lloyd E. K., Wilson R. J. (1986). *Graph Theory, 1736-1936*.

[18] Mao X. R. (2007). *Stochastic Differential Equations and Application*.

[19] Lai Y. C., Park K. (2006). Noise-sensitive measure for stochastic resonance in biological oscillators. *Mathematical Biosciences and Engineering*.

[20] Zuparic M. L., Kalloniatis A. C. (2013). Stochastic (in)stability of synchronisation of oscillators on networks. *Physica D: Nonlinear Phenomena*.

[21] Zhang C., Li W., Wang K. (2017). Exponential synchronization of stochastic coupled oscillators networks with delays. *Applicable Analysis*.

[22] Li S., Su H., Ding X. (2018). Synchronized stationary distribution of hybrid stochastic coupled systems with applications to coupled oscillators and a Chua’s circuits network. *Journal of the Franklin Institute*.

